# The Hippo transducer TAZ promotes cell proliferation and tumor formation of glioblastoma cells through EGFR pathway

**DOI:** 10.18632/oncotarget.9199

**Published:** 2016-05-06

**Authors:** Rui Yang, Yanan Wu, Jiahua Zou, Ji Zhou, Mei Wang, Xiangwei Hao, Hongjuan Cui

**Affiliations:** ^1^ State Key Laboratory of Silkworm Genome Biology, Southwest University, Chongqing 400715, China; ^2^ Department of Neurosurgery, Second Artillery General Hospital, Chinese People's Liberation Army, Beijing 100088, China; ^3^ Chongqing Reproductive and Genentics Institute, Chongqing Obstetrics and Gynecology Hospital, Chongqing 400013, China

**Keywords:** TAZ, glioblastoma, cell proliferation, cell cycle, EGFR

## Abstract

TAZ, a WW-domain-containing transcriptional co-activator, is important for development of various tissues in mammals. Recently, TAZ has been found to be overexpressed in some types of human cancers. However, the role of TAZ in glioblastoma remains unclear. In this study, we found that TAZ was overexpressed in prognostically poor glioblastoma patients. Through knocking down or overexpressing TAZ in U87 and LN229 cells, the expression level of TAZ was found to be positively related to cell proliferation *in vitro* and tumor formation *in vivo*. Further investigation indicated that TAZ could significantly promote the acceleration of cell cycle. Moreover, the western blot for p-EGFR, p-AKT, p-ERK1/2, p21, cyclin E and CDK2 proteins, target genes of the EGFR pathway, indicated that TAZ significantly activated EGFR/AKT/ERK signaling. Additionally, the blockage of EGFR pathway resulted in a significantly inhibition of cell proliferation induced by TAZ. Taken together, these results demonstrate that TAZ can promote proliferation and tumor formation in glioblastoma cells by potentiating the EGFR/AKT/ERK pathway, and provide the evidence for promising target for the treatment of glioblastoma.

## INTRODUCTION

Glioblastoma (GBM) is a common and primary brain tumor, with poor prognosis and few therapeutic advances in the last decade. The median survival of GBM patients is only about 15 months [1–3]. The genetic, bacterial virulence, environmental, and other factors have been in regulating the GBM process, but the molecular mechanism is weakly understood [4]. Therefore, better defining the pathogenesis of GBM, exploring biomarkers, and finding novel targets for treatment are urgently demanding.

TAZ, also known as WWTR1, which is a WW-domain-containing transcriptional co-activator, is important for development of many tissues in mammals [5, 6]. TAZ could bind with many transcription factors such as the RUNX family, Pax3, TBX5, TIF-1 and READ [7–9]. Recently, TAZ was identified as a component of Hippo-LATS pathway, which is participated in transcriptional outcome to promote cell proliferation and inhibit apoptosis [10]. Most recently, enhanced expression of TAZ has been found in many malignant tumors, including gastric cancer, oral cancer, non-small cell lung cancer (NSCLC), breast cancer and neuroblastoma [11–14]. Overexpression of TAZ has been shown to promote cell proliferation and tumorigenesis in breast cancer, neuroblastoma and NSCLC cells, whereas knocking down TAZ expression suppresses cell proliferation and tumor formation, suggesting that TAZ may function as an oncogene in breast cancer, NSCLC and neuroblastoma. In glioma, TAZ could regulate mesenchymal differentiation and tumor invasion [15]. However, the role of TAZ in regulating tumor progression in glioblastoma cells has not been explored.

The frequent amplification of the epidermal growth factor receptor (EGFR) in GBM was firstly reported in 1985 and it has been confirmed in many subsequent studies [16]. According to statistics, the EGFR gene is amplified in 30%–40% of GBM patients, and nearly 50% of them highly express the receptor [1]. EGFR is a member of ErbB family, which is activated by phosphorylating the tyrosine kinase moiety [17, 18]. Following EGFR activation, three pathways are activated, including the PI3K/AKT kinase pathway, the Ras-ERK cascade, and the STAT3-dependent signaling events [1, 19–22]. EGFR activation accelerates cell cycle progression, supports differentiation and migration, and inhibits apoptosis [22–25]. In GBM cells, EGFR activation promote cancer cell growth and survival, inhibition of EGFR slows cell migration [26–28]. Ninov N *et al.* reported that activation of EGFR pathway could increase the expression of cyclin E and CDK2 and then accelerate cell cycle progression [28]. There was evidence that TAZ also was involved in EGFR pathway in the regulation of cell proliferation [29]. Therefore, we hypothesized that TAZ might also contribute to GBM cell proliferation and tumor formation through EGFR pathway.

In this study, we provided the evidence that overexpression of TAZ induced cell proliferation and tumorigenicity in glioblastoma, whereas knockdown of TAZ inhibited cell proliferation and tumorigenicity in glioblastoma. Mechanistically, we found that TAZ promoted cell proliferation and tumor formation of GBM cells by potentiating the EGFR/AKT/ERK pathway, whereas all the effects were blocked by the EGFR inhibitor Erlotinib. Taken together, our findings demonstrate that TAZ promotes glioblastoma growth through the EGFR/AKT/ERK pathway, and provide the evidence for promising target for the treatment of glioblastoma.

## RESULTS

### High expression of TAZ correlates with poor patient prognosis

To determine whether alterations at the genetic locus of TAZ could be implicated in GBM patient prognosis, survival data from R2 genomics analysis and visualization platform database were used to evaluate the effects of TAZ on overall patient survival. TAZ was highly expressed in 104 out of 504 cases of glioblastoma, and high expression very significantly correlated with reduced patient survival in TCGA's data, *p* = 7.8e–0.5 (Figure 1A). Similarly, in Frence data set consisting of 284 patients, there were 122 cases with upregulation TAZ, also confirmed that high level of TAZ was associated with poor prognosis, *p* = 4.5e–11 (Figure 1B). Accordingly, contrasting to normal tissue or low grade astrocytoma, TAZ was significantly upregulated in GBM patients according to TCGA's data, French's data and sun's date (Figure 1C, 1D and 1E). To further confirm the TAZ expression results in GBM, a western blot assay was used to measure the GBM cell lines, tissues derived from normal tissue, tumor center and peritumor, the result revealed that TAZ was commonly expressed in GBM cell lines (U118, U251 LN229, A172 and U87) and highly expressed in tumor center compared to normal tissue. All these results indicated that TAZ might function as an oncogene involved in the development and progression of GBM.

**Figure 1:** High TAZ expression is a prognostic indicator of poor survival in glioblastoma patients (**A**) Kaplan-Meier analysis of progression-free survival for the TCGA database with the log rank test *P* value was indicated. Cutoff:400-1094.1: raw p: 4.4e-5 (bonf: 0.021) (**B**) Kaplan-Meier analysis of progression-free survival for the Frence database with the log rank test *P* value indicated. Cutoff: 151-1028.0: raw p: 1.4e-11 (bonf: 3.6e-09) (**C**) Box plot of TAZ expression levels from non-tumor, GBM and recurrent GBM patients was shown. (**D**) Box plot of TAZ expression levels in the normal, stage 1 to 3 and GBM tumors. (**E**) Box plot of TAZ expression levels in the stage 2 and 4 tumors. (**F**) Western blot assay of TAZ expression in GBM cell lines and different tissues was performed. All data are shown as the mean ± SD, *p < 0.05, **p < 0.01. All *p* values are based on analysis control versus treatment.

### TAZ is essential for proliferation of GBM cells

To test the effects of TAZ expression in cell proliferation and growth, stable TAZ-knockdown cells (U87-shTAZ and LN229-shTAZ) and stable TAZ-overexpressing cells (U87-TAZ and LN229-TAZ) were established. Western blot analysis showed that the TAZ was effectively down-regulated or overexpressed respectively (Figure 2A and 2D). Next, the proliferation kinetics of GBM cells was investigated via cell growth curve and MTT assay. The growth curve (Figure 2B, 2E) revealed that TAZ knockdown in both U87 (Figure 2B) and LN229 (Figure 2E) cells resulted in a significant growth inhibition. However, TAZ overexpression markedly promoted cell growth (Figure 2B and 2E). Furthermore, MTT assays with U87 and LN229 cells confirmed that TAZ knockdown resulted in a significant inhibition in cell viability and that TAZ overexpression led to a marked increase in cell viability (Figure 2C and 2F). Above data were confirmed by BrdU incorporation in the U87 and LN229 cell lines, where the TAZ-knockdown cells showed over a 40% reduction, while the TAZ-overexpressing cells showed over a 70% increment in DNA synthesis compared to control cells in the two cell lines (Figure 2G and 2H). These results demonstrated that TAZ was essential for proliferation of GBM cells.

**Figure 2:** TAZ promotes GBM cell growth and proliferation (**A**) Western blot assay was used to characterize the expression of TAZ in TAZ-knockdown U87 cells and TAZ-overexpressing U87 cells. (**B**) The effect of TAZ on the proliferation of U87 cells. (**C**) The effect of TAZ on the viability of U87 cells. (**D**) Western blot assay was used to characterize the expression of TAZ in TAZ-knockdown LN229 cells and TAZ-overexpressing LN229 cells. (**E**) The effect of TAZ on the proliferation of LN229 cells. (**F**) The effect of TAZ on the viability of LN229 cells. (**G, H**) Image and quantification of U87 and LN229 cells positive for BrdU staining. All data are shown as the mean ± SD, *p < 0.05, **p < 0.01. All *p* values are based on analysis control versus treatment.

### TAZ promotes colony formation *in vitro* and tumor formation of GBM cells *in vivo*

To further uncover the effects of TAZ expression in colony formation, soft agar assay was employed *in vitro*. As shown in Figure 3A and 3B, the colonies were smaller and lesser in TAZ-knockdown cells compared with the controls. However, those were bigger and more in TAZ-overexpressing cells. Xenograft experiment showed that the tumors formed by the TAZ-knockdown U87 cells grew much slower (Figure 3C). And those formed by the TAZ-overexpressing U87 cells grew much faster (Figure 3D). At the termination of the experiment, the mice were sacrificed, and the tumors were excised. The volume of tumors formed by TAZ-knockdown cells was smaller, while those formed by TAZ-overexpressing U87 cells were greater (Figure 3C and 3D). These results indicated that TAZ could promote the tumor growth of GBM cells. To determine whether TAZ enhances the tumor progress of GBM cells by accelerating cell proliferation, a widely known cell proliferation marker-Ki67, was tested in the tumor xenografts tissues by immunohistochemical staining. The expression of Ki67 in the tumor tissues formed by the TAZ-knockdown U87 cells was decreased compared with the shCtr cells (Figure 3E and 3F). The results suggested that TAZ most likely enhanced the tumor progression of GBM cells by accelerating cell proliferation.

**Figure 3:** TAZ promotes colony formation and tumor formation of U87 cells in immunodeficient mice (**A, B**) The effects of TAZ on the colony formation in TAZ-knockdown U87 cells and TAZ-overexpressing U87 cells. (**C**) The tumor growth curve of TAZ-knockdown U87 cells injected into immunodeficient mice. (**D**) The tumor growth curve of TAZ-overexpressing U87 cells injected into immunodeficient mice. (**E**) Immunohistochemical staining for Ki67 in tumor tissues, shTAZ: shRNA for TAZ; shCtr: shRNA for control. Values are shown as the mean ± SD. *p < 0.05, **p < 0.01. All *p* values are based on analysis control versus treatment.

### TAZ accelerates cell cycle progression in GBM cells

Since cell multiplication change usually involves adjustment of the cell cycle, the U87 and LN229 cell cycle was analyzed by flow cytometry to examine whether TAZ promotes cell multiplication by accelerating the cell cycle progress. Representative histograms and the results are summarized in Figure 4A–4D. TAZ knockdown resulted in a marked increase in the percentage of both U87 and LN229 cells in G1 phase. Conversely, TAZ overexpression significantly decrease the G1 phase percentage both cell types. To confirm the results, we measured the expression of cyclin E2, CDK2 and p21 which could impress cells to pass the G1/S checkpoint. Knockdown TAZ downregulated the level of cyclin E2 and CDK2 as well as increased the protein level of the CDK2 inhibitor p21. Whereas overexpressing TAZ increased the expression of cyclin E2 and CDK2 as well as downregulated the level of p21 (Figure 4E–4H). These results suggested that TAZ accelerated cell cycle progression by upregulating of the CCNE2-CDK2 complex.

**Figure 4:** TAZ accelerates the cell cycle in GBM cells (**A**) The cell cycle of TAZ-modulated U87 cells was analyzed by flow cytometry. (**B**) The effect of TAZ on the cell cycle of U87 cells. (**C**) The cell cycle of TAZ-modulated LN229 cells was analyzed by flow cytometry. (**D**) The effect of TAZ on the cell cycle of LN229 cells. (**E, G**) Western blot analysis of cyclin E2, CDK2 and p21 expression in TAZ-modulated cells; representative blots are shown. (**F, H**) Quantitative analysis of cyclins and CDKs expression in TAZ-modulated cells; GAPDH was used as a loading control; student's *t*-test was carried out. All data are shown as the mean ± SD, *p < 0.05, **p < 0.01.

### TAZ potentiates the EGFR pathway in GBM

It has been reported that activating of the EGFR, the epidermal growth factor receptor, could accelerate cell cycle progression by activating the cyclin E-CDK2 kinase, and then promote cell proliferation. EGFR is a crucial signaling molecule, and Ras-ERK and PI3K/AKT are important downstream pathways of EGFR. Therefore, the expression of p-EGFR, p-AKT and p-ERK1/2 proteins was measured by western blot assay in shCtr, TAZ-knockdown, vector and TAZ-overexpressing GBM cells. Representative blots for U87 and LN229 cells and the results are summarized are shown in Figure 5A–5D. To test whether the expression of TAZ is also associated with EGFR signaling *in vivo*, the expression of the p-EGFR, p-AKT and p-ERK1/2 proteins was examined in the xenograft tumor tissues formed by TAZ-knockdown and TAZ-overexpressing U87 cells (Figure 5E and 5F). The expression of these proteins in TAZ-knockdown cells and in the tumor tissues formed by the TAZ-knockdown U87 cells was all markedly reduced compared with their controls. Whereas that in TAZ-overexpressing cells and in the tumor tissues formed by the TAZ-overexpressing U87 cells was all significantly increased compared with their controls. All these results indicated that the TAZ-promoted proliferation and tumor formation of GBM cells were possibly mediated by potentiating the EGFR signaling pathway.

**Figure 5:** TAZ enhances the activity of the EGFR/AKT/ERK pathway (**A**) The expression of p-EGFR, EGFR, p-AKT, AKT, p-ERK1/2 and ERK1/2 in TAZ-modulated U87 cells was measured by western blot assay. (**B**) The quantitative analysis of p-EGFR, p-AKT, p-ERK1/2 relative expression in TAZ-modulated U87 cells. (**C**) The expression of p-EGFR, EGFR, p-AKT, AKT, p-ERK1/2 and ERK1/2 in TAZ-modulated LN229 cells was measured by western blot assay. (**D**) The quantitative analysis of p-EGFR, p-AKT, p-ERK1/2 relative expressions in TAZ-modulated LN229 cells. (**E**) The expression of p-EGFR, EGFR, p-AKT, AKT, p-ERK1/2 and ERK1/2 in tumor xenografts was measured by western blot. (**F**) The quantitative analysis of p-EGFR, p-AKT, p-ERK1/2 relative expressions in tumor xenografts. All data are shown as the mean ± SD, *p < 0.05, **p < 0.01.

### Blockage of the EGFR/AKT/ERK pathway by erlotinib attenuates the cell proliferation mediated by TAZ expression

Erlotinib is a novel, oral, highly selective tyrosine kinase inhibitor of the EGFR. To further confirm that TAZ promotes the proliferation by potentiating the EGFR pathway, erlotinib was used to inhibit the EGFR in TAZ-modulated GBM cells. The phosphorylation levels of EGFR, AKT and ERK1/2 in the erlotinib-treated, TAZ-overexpressing GBM cells were significantly decreased compared to those in the cells without erlotinib treatment (Figure 6A, 6B, 6D, and 6E). This result suggested that erlotinib treatment eliminated the potentiation of the EGFR pathway by TAZ, indicating that TAZ indeed influences the activity of the EGFR pathway. While treatment with erlotinib resulted in no remarkable increase in the expression of TAZ in TAZ-overexpressing GBM cells (Figure 6A, 6B, 6D, and 6E). It indicated that TAZ is the upstream of the EGFR. Consistent with the observations above, erlotinib treatment resulted in a significant inhibition in cell proliferation and viability in the TAZ-overexpressing GBM cells (Figure 6C and 6F), indicating that erlotinib can arrest the cell proliferation and viability induced by TAZ. Taken together, these results demonstrated that the TAZ-mediated promotion of GBM cell proliferation is mediated by the EGFR pathway.

**Figure 6:** Erlotinib treatment attenuates the increasing proliferation of GBM cells induced by TAZ TAZ-modulated U87 and LN229 cells were treated with the EGFR inhibitor erlotinib (0.1 μM), and the expression of p-EGFR, p-AKT, and p-ERK1/2 was measured by western blot. (**A, B**) The representative blot and quantitative analysis of p-EGFR, EGFR, p-AKT, AKT, p-ERK1/2 and ERK1/2 expression in U87 cells were shown. (**C**) The effect of erlotinib on the viability of TAZ-modulated U87 cells was measured by the MTT assay. (**D, E**) The representative blot and quantitative analysis of p-EGFR, EGFR, p-AKT, AKT, p-ERK1/2 and ERK1/2 expression in LN229 cells were shown. (**F**) The effect of erlotinib on the viability of TAZ-modulated LN229 cells was measured by the MTT assay. Values are shown as the mean ± SD. *p < 0.05, **p < 0.01. All *p* values are based on analysis control versus treatment.

## DISCUSSION

TAZ, a WW-domain-containing transcriptional co-activator, which is important for development of various tissues in mammals. In recent years, enhanced expression of TAZ has been found in many malignant tumors, including gastric cancer, breast cancer, oral cancer, non-small cell lung cancer (NSCLC) and neuroblastoma, suggesting that TAZ is important for tumorigenesis [10–14]. In glioma, TAZ could regulate mesenchymal differentiation and tumor invasion [15]. However, the role of TAZ in regulating cell proliferation and tumor formation in glioblastoma cells has not been explored. We first evaluated the clinical significance of TAZ in a large cohort of GBM patients and found a negative association of TAZ expression with overall survival. Furthermore, we found that TAZ protein levels were significantly elevated in the tumor tissue over normal in GBM sample, suggesting that TAZ may promote the development and progression of GBM.

Subsequently, through shRNA knockdown or stable plasmid transfection, the TAZ protein level was found to be positively related to the proliferation of GBM cells. Tumor xenograft experiments in nude mice indicated that TAZ significantly promoted glioma growth *in vivo*. Moreover, immunostaining assays revealed that tumor tissues formed by TAZ-overexpressing cells had much stronger Ki67 expression, suggesting that TAZ promoted the tumor formation of GBM cells by accelerating cell proliferation. Furthermore, a cell cycle analysis by FACS revealed that increased TAZ expression resulted in a significant decrease in the percentage of G0/G1 phase cells, suggesting that TAZ accelerates the cell cycle in GBM cells. All of our findings together indicate that TAZ functions to promote the development and progression of GBM, consistent with previous reports in gastric cancer, breast cancer, oral cancer, non-small cell lung cancer (NSCLC) and neuroblastoma.

Recently, TAZ was found to potentiate EGFR signaling in MCF10A cells and play important roles in breast tumor growth and metastasis [30]. EGFR was highly expressed in GBM cells; the activation of EGFR could accelerate cell cycle progression and promote cell proliferation by activating its downstream signaling pathway (PI3K/AKT and Ras-ERK) [18, 19]. In our previous study, we found that TAZ functions as a receptor of HDAC9 to enhance EGFR phosphorylation, and then activate EGFR/AKT/ERK signaling [31]. In the present study, TAZ was found to potentiated EGFR and its downstream signaling pathways activation in GBM cells and xenograft tumors. These results suggest that TAZ activate EGFR pathway in GBM cells. Ninov N *et al.* reported that activation of EGFR pathway could increase the expression of cyclin E and CDK2 and then accelerate cell cycle progression [28]. TAZ might regulate cell cycle and cell cycle proteins not directly, but by potentiating the EGFR/AKT/ERK pathway.

An increasing number of studies have demonstrated that TAZ promotes tumorigenesis, accelerates cell proliferation, and activates the EGFR pathway. However, it remains inconclusive whether TAZ promotes cell proliferation and tumorigenesis by activating EGFR pathway. TAZ, as a transcriptional regulator rather than a kinase, activates EGFR signal but not up-regulates EGFR. This observation actually suggests a possibility for an indirect process for activation of EGFR by TAZ, TAZ might transcriptionally induce expression of some other factors (e.g., ligands of EGFR) that in turn result in EGFR activation. Yang Nuo et al. demonstrated a EGFR ligand amphiregulin is a target of TAZ [30]. Therefore, TAZ might transcriptionally induce expression of AREG that in turn result in EGFR activation. In the present study, blockage with Erlotinib, an inhibitor of EGFR activation, resulted in a significant inhibition of the GBM cell proliferation induced by TAZ, suggesting that TAZ promotes GBM cell proliferation via activation of EGFR pathway.

In summary, our study demonstrates that TAZ promotes cell proliferation and tumor formation in GBM cells by activating the EGFR/AKT/ERK pathway. Therefore, we propose a hypothesis in which TAZ potentiates EGFR signaling, accelerates the cell cycle, and promotes cell proliferation, eventually leading to the progression of glioblastoma. Our study indicates that TAZ could be a novel and promising target for glioblastoma treatment.

## MATERIALS AND METHODS

### Cell lines and cell culture

Human glioblastoma cell lines (U87, LN229 and A172) were purchased from American Type Culture Collection (ATCC, Rockville, MD, USA). All the cells were cultured in DMEM (Invitrogen) supplemented with 10% fetal bovine serum, 2 nM L-glutamine, 100 U/ml penicillin and 0.1 mg/ml streptomycin. All cells were maintained in a humidified atmosphere containing 5% CO2 at 37°C.

### Reagents

Erlotinib (Santa Cruz) was dissolved in Dimethy1 Sulfoxide (DMSO). Mouse monoclonal anti-TAZ, anti-cyclin E2, anti-CDK2 and anti-GAPDH were obtained from Santa Cruz. Rabbit monoclonal anti-EGFR, anti-phospho-EGFR, anti-AKT, anti-phospho-EGFR, anti-ERK1/2, anti-phospho-ERK1/2 and anti-p21 were obtain from Cell Signaling Technology. Mouse monoclonal anti-Ki67 and propidium iodide (PI) were obtained from BD Biosciences.

### Vector construction, transfection and infection

The small interfering RNA expression vector that expresses TAZ-specific short hairpin RNA (shTAZ), TAZ-specific short hairpin RNA (shTAZ) and negative control (shCtr) were purchased from GenePharma Co., Ltd (Shanghai, China). Human fulllength TAZ cDNA was obtain from Queen's University Richardon Lab, the DNA fragment was subsequently cloned into pCDH-CMV-MCS-EF1-puro vector to generate the recombinant plasmid [32]. The TAZ shRNA, TAZ shRNA and TAZ overexpression vectors were transfected into 293FT cells using the Lipofectamine 2000 reagent (Invitrogen, Carlsbad, CA, USA) according to the manufacturer's protocol, and then the Lentivirus were infected into GBM cells. The transfected cells were selected with puromysin for 1 week, and drug-resistant cells were collected, expanded and identified.

### Cell proliferation and viability assays

Cells were seeded and cultured in 6-well plates at the concentration of 1 × 10^5^ cells/well. The cells were harvested and counted daily for 5 days using a hemocytometer, and cell proliferation was assessed by cell growth curves. To test cell viability, 1 × 10^3^ cells were cultured in 96-well plates for 5 days, and MTT assay was performed according to the manufacturer's protocol. All experiments were performed independently in triplicate.

### BrdU staining

For BrdU immunofluorescent staining, cells were grown on coverslips, and incubated with 10 μg/ml BrdU (Sigma) for 30 min, then washed with phosphate buffered saline (PBS) and fixed in 4% paraformaldehyde (PFA) for 20 min. Subsequently, cells were pre-treated with 1 mol/L HCl, and blocked with 10% goat serum for 1 h, followed by a monoclonal rat primary antibody against BrdU (1:200, ab6326, Abcam, Cambridge, MA, USA) for 1 h and Alexa FluorR^®^ 594 goat anti-rat IgG secondary antibody, (H + L; Invitrogen). DAPI (300 nM) was used for nuclear staining; the percentage of BrdU was calculated at least from 10 microscopic fields (Nikon 80i, Nikon Corporation, Tokyo, Japan).

### Soft agar assay

In total, 1 × 10^3^ cells were mixed with 0.3% Noble agar in growth medium and plated into six-well plates containing a solidified bottom layer (0.6% Noble agar in growth medium). The colonies were photographed after 14 to 21 days and recorded.

### Animal studies

Animal experiments were performed in the compliance with the guidelines of the Institute for Laboratory Animal Research, Southwest University. Five- to 6 -week-old male nude mice were used in the experiments. Subcuticular injections were performed following a previous protocol with minor modifications [31]. Briefly, U87-shCtr (1×10^6^ cells in 100 μl of PBS) was inoculated subcutaneously into the right flank of nude mice and U87-shTAZ was inoculated subcutaneously into the left flank. Similarly, U87-vector and U87-TAZ cells were inoculated subcutaneously into the nude mice. The tumor size was measured using a vernier caliper every week, and the volume was calculated with the following formula: V = (length × width^2^)/2. At the termination of the experiment, the tumor mass was harvested, weighed, and stored for immunostaining or protein extract.

### Flow cytometry

For cell cycle analysis, 1 × 10^6^ cells were harvested and washed twice with cold PBS, followed by fixation with ice-cold 70% ethanol overnight at 4°C. After washing twice with PBS, the cells were incubated with propidium iodide (PI) (BD Biosciences, San Jose, CA, USA) and RNaseA for 30 min at room temperature. The cells were then analyzed using a FACS C6 (BD Biosciences, San Jose, CA, USA) with CellQuest software.

### Western blot

Cells were lysed in a lysis buffer containing 50 mM Tris-HCl, pH 7.5, 150 mM NaCl, 1% Nonidet P-40, 0.25% sodium deoxycholate, 0.1% SDS with complete protease inhibitor cocktail (Roche) and phosphatase inhibitors (Sigma-Aldrich). Cell lysates were separated by 10% SDSPAGE and were transferred to a polyvinylidene difluoride membrane. SDSPAGE gels were calibrated using Magic Mark XP Western Standard (Invitrogen). Primary antibodies were used at a dilution of 1:1,000. Secondary antibodies (peroxidase-labeled anti-mouse and anti-rabbit antibodies) were used at a dilution of 1:5,000. Bound antibodies were visualized by chemiluminescence using the ECL Prime Western blotting (WB) detection system (GE Healthcare), and luminescent images were analyzed with a Lumino Imager (LAS- 4000 mini; Fuji Film Inc.).

### Immunohistochemistry staining

Paraffin embedded tumor tissues were sectioned at 5 μm, deparaffinized, and rehydrated. For antigen retrieval, sections were treated for 20 minutes at 95°C in 10 mmol/L citrate buffer (pH 6.0) in a laboratory microwave oven and subsequently washed in PBS. For immunohistochemistry, after quenching of endogenous peroxidase activity and blocking with normal goat serum, sections were incubated sequentially with Ki67 primary antibodies (1:100, clone 550609, BD pharmingen), biotinylated goat anti-mouse IgG, and the ABC reagent (Vector Laboratories). The immunostaining was visualized with 3, 3′-diaminobenzidine (Sigma). Sections were then counterstained with hematoxylin before being examined using a light microscope.

### Patient data analysis

Patient data and gene expression datasets were obtained from R2: microarray analysis and visualization platform (http://hgserver1.amc.nl/cgi-bin/r2/main.cgi). All prognosis analyses were conducted online, and all data and *P* values (log-rank test) were downloaded. Kaplan– Meier analysis and the resulting survival curves were performed using GraphPad Prism (version 6.0). All cutoff values for separating high and low expression groups were determined by the online R2 database algorithm.

### Statistical analysis

All observations were confirmed by at least three independent experiments. Quantitative data are expressed as the mean ± standard deviation. Two-tailed Student's *t*-test was performed for paired samples. *P* < 0.05 was considered statistically significant.
